# Clinical Features and Risk Factors of Fever in Acute Gouty Arthritis

**DOI:** 10.1155/2022/8798838

**Published:** 2022-10-03

**Authors:** Yan Huang, Meiju Zhou, Fang Yuan

**Affiliations:** Department of Rheumatology and Immunology, Zhejiang Hospital, 1229 Gudun Road, Xihu District, Hangzhou, Zhejiang Province 310030, China

## Abstract

**Objectives:**

This study aimed to investigate the clinical characteristics and risk factors of fever in hospitalised patients with acute gouty arthritis (AGA).

**Methods:**

The clinical data of 167 hospitalised patients with AGA who met the inclusion criteria were retrospectively analysed. The demographic, clinical, and medication data of patients with and without fever were compared, and risk factors associated with fever were identified via logistic regression analysis.

**Results:**

The incidence of fever in hospitalised patients with AGA was 31.1%, with low-grade fever being predominant. Visual analogue scale (VAS) scores, white blood cell counts, neutrophil proportion, C-reactive protein (CRP) levels, and erythrocyte sedimentation rate (ESR) were higher in the fever group than in the non-fever group (*P* < 0.05 for all). In addition, the incidence rates of arthritis of single knee and polyarthritis were higher in patients in the fever group (*P* < 0.05). The proportion of patients who received betamethasone injection and combination therapy were higher in the fever group (*P* < 0.05). However, no significant differences were observed in age; sex; uric acid (UA) levels; and the incidence rate of hypertension, diabetes mellitus, cardiovascular disease, and renal function abnormalities between the two groups. Logistic regression analysis revealed that arthritis of single knee, polyarthritis, age of ≥65 years, CRP levels, and VAS scores were risk factors for concomitant AGA and fever. Among these factors, CRP levels and VAS scores were identified as independent risk factors (odds ratio [OR], 1.014 and 1.686, respectively; 95% confidence interval [CI], 1.004–1.025 and 1.115–2.549, respectively; *P* < 0.05 for both).

**Conclusion:**

The incidence of fever is high in hospitalised patients with AGA. Elderly patients, patients with arthritis affecting only one knee, and those with polyarthritis are predisposed to fever. In addition, the risk of developing fever increases with increasing VAS scores and CRP levels, and patients presenting with fever require enhanced anti-inflammatory and analgesic therapy.

## 1. Introduction

Gout, a metabolic rheumatic disease, has a prevalence of 0.03–15.3% among different races [1]. Gout arthritis (GA) is an inflammatory joint disease caused by the accumulation of uric acid (UA) in the synovium, bone, joint capsule, cartilage, and tissues. The symptoms of GA include swollen and painful joints, elevated local skin temperature, dysfunction of activity, and fever [2, 3]. Low-grade fever is predominant [2], whereas high-grade fever is occasionally observed [4]. The clinical manifestations of acute gouty arthritis with fever (AGA–fever) are similar to those of infective fever; therefore, both conditions are indistinguishable. Patients with fever are required to first visit a fever clinic and undergo routine screening for COVID-19 infection, which increases their psychological burden. In clinical practice, patients with lower-extremity joint swelling and pain accompanied by fever and hyperuricemia are often treated with antibiotics, especially in the fever clinic and emergency department. Clinical signs including fever; elevation of inflammation-related parameters; joint pain caused by infectious arthritis; and noninfectious causes of inflammation, such as gout, should be considered for differential diagnosis. At present, the clinical characteristics and risk factors of AGA–fever remain elusive. In this study, the clinical characteristics and risk factors of AGA–fever were investigated by comparing the data of patients with and without fever, who did not have pathogenic and imaging evidence of infection and had not received antibiotic treatment. This study provides insights into the clinical treatment of AGA–fever and suggests that the unnecessary use of antibiotics should be reduced.

## 2. Material and Methods

### 2.1. Study Participants

Patients who were hospitalised in Zhejiang Hospital from April 2019 to November 2020 were initially selected. The inclusion criteria were as follows [5]: (1) patients aged ≥18 years; (2) patients fulfilling the 2015 ACR/EULAR gout classification diagnostic criteria [5]^;^ (3) patients with VAS scores of ≥1 for joint pain; (4) patients who did not exhibit infection-related signs and symptoms, have pathogenic and imaging evidence of infection, and receive antibiotic treatment; (5) patients in whom the use of adequate nonsteroidal anti-inflammatory drugs (NSAIDs) or hormone therapy reduced the body temperature to normal within 24 hours. The exclusion criteria were as follows: (1) patients who did not meet the diagnostic criteria for gout; (2) patients aged <18 years; (3) patients with secondary gout; (4) patients with concurrent infectious diseases such as pulmonary, gastrointestinal, urinary tract, skin, or soft tissue infections; (5) patients with concurrent rheumatic immune diseases such as ankylosing spondylitis, rheumatoid arthritis, and systemic lupus erythematosus; (6) patients with concurrent hyperthyroidism; and (7) patients receiving antibiotics. Eventually, a total of 167 patients were included in the study. This study was approved by the Ethics Committee of Zhejiang Hospital (approval No: 2021; 112 K).

### 2.2. Research Methodology

Patient data, including the body temperature, sex, age, duration of disease, VAS scores, and the type and involved joints, were obtained. The duration of gout was defined as the time between the occurrence of the first gout symptom and the present visit to the hospital. ≥3 joints involvement indicated polyarthritis (the knee joint was not considered an involved site in polyarthritis). Patients were classified based on age into the young and middle-aged (from 18 to <65 years) and elderly (≥65 years) groups, which is similar to age classification methods used in previous studies [6, 7]. In addition, procalcitonin (PCT) levels, UA levels, white blood cell count, neutrophil proportion, erythrocyte sedimentation rate (ESR), C-reactive protein (CRP) levels, and medication used were evaluated in all patients. Eventually, patients were divided into the fever (*n* = 52) and non-fever (*n* = 115) groups according to the threshold temperature of 37.3°C.

### 2.3. Statistical Analysis

The SPSS Statistics (version 22.0) software was used for statistical analysis. Measurement data conforming to normal distribution were expressed as mean ± standard deviation (x̅±s), and a *t*-test was used for comparing data between two groups. Measurement data not conforming to normal distribution were expressed as the median (quartile) M (Q1, Q3), and Mann–Whitney *U* rank-sum test was used for comparing data between two groups. Categorical variables were expressed as a percentage (%), and the chi-square test was used for data comparison. In addition, univariate logistic regression analysis was performed to determine the influencing factors of AGA–fever, and binary logistic regression analysis was performed based on UA levels and variables with *P* values of ≤0.1. A *P* value of <0.05 indicated significant differences.

## 3. Results

### 3.1. General Information

In this study, a total of 190 patients with AGA are hospitalised in Zhejiang Hospital from April 2019 to November 2020 were initially selected; of which, 167 were included after excluding 23 patients who had incomplete clinical data and did not meet the inclusion criteria. Of the 167 patients, 154 (92.2%) were men, with a median age of 58 (38, 70) years and a median disease duration of 5 (3, 10) years. In addition, 31.1% (52/167) of patients developed a fever (low-grade fever, 37.3–38°C; moderate-grade fever, 38.1–39°C; and high-grade fever, >39.1°C). The number of low-grade fever cases was highest, whereas that of high-grade fever was lowest. PCT levels were normal (<0.5*u*g/L) in all patients with fever (Table 1).

### 3.2. Clinical Data

White blood cell counts, neutrophil proportion, VAS scores, ESR, and CRP levels were higher in the fever group than in the non-fever group (*P* < 0.05). However, no significant differences were observed in age; sex; disease course; UA indicators, and the incidence rates of hypertension, diabetes mellitus, cardiovascular diseases, and renal function abnormalities between the two groups (*P* > 0.05). The proportion of patients who received betamethasone injection and combination with NSAIDs therapy was higher in the fever group than in the non-fever group (*P* < 0.05). However, no significant differences were observed in the proportion of patients who received colchicine, NSAID, and oral hormone therapy between the two groups. The proportion of patients' age of ≥65 years in the fever group was higher than in the non-fever group (*P* < 0.05) (Table 2).

### 3.3. Comparison of Involved Sites

The proportion of patients with arthritis of single knee and polyarthritis was higher in the fever group than in the non-fever group (the knee joint was not considered an involvement site in polyarthritis). In addition, the proportion of patients with pain in the first toe joint was lower in the fever group than in the non-fever group (*P* < 0.05). However, no significant differences were observed among other involved sites (*P* > 0.05 for all). Univariate analysis suggested that arthritis affecting only one knee and polyarthritis were risk factors for AGA–fever (Table 3 and Figure 1).

### 3.4. Multivariate Analysis

White blood cell counts, neutrophil proportion, CRP levels, ESR, age of ≥65 years, VAS scores, UA levels, arthritis of a single knee, and polyarthritis were selected as variables for multivariate logistic regression analysis. The results revealed that elevated CRP levels and VAS scores were independent risk factors for AGA–fever (Table 4 and Figure 2).

## 4. Discussion

The incidence of gout is increasing worldwide [8]. At present, gout is the second most common disease after diabetes mellitus [9]. AGA is characterised by inflammation caused by the accumulation of monosodium urate (MSU) in the joints and tissues. It is known as the “king of pain” [10]. A few patients with gout have transient fever, elevated white blood cell counts [3], and rarely, persistent fever [11]. Concomitant gout and fever cannot be easily distinguished from infective diseases. This study aimed to analyse the risk factors of AGA–fever and provide a reference for its clinical treatment.

In this study, low-grade fever was found to be predominant among patients with AGA, whereas high-grade fever was the least common. PCT levels were normal in all patients with AGA–fever. In addition, white blood cell counts, neutrophil proportion, ESR, CRP levels, and VAS scores were significantly higher among patients with fever than among those without fever. These results suggest that patients with AGA–fever have a more intense inflammatory response and higher pain levels than patients without fever. Drugs used for the treatment of AGA include colchicine, NSAIDs, and glucocorticoids [12]. Glucocorticoids, such as injectable betamethasone, are used as second-line agents. In this study, the proportion of patients who received betamethasone injection or combination NSAID therapy was higher in the fever group than in the non-fever group, indicating that stronger anti-inflammatory and analgesic drugs should be recommended for patients with AGA–fever. Therefore, AGA with symptoms of fever can serve as a predictor of refractory gout.

Inflammation in gout is attributed to the activation of white blood cells by MSU, leading to the production of various cytokines [13]. Gout mostly occurs in lower-extremity joints [14]. In this study, 38.5% of patients had single-knee-joint involvement and 21.2% of patients had multiple-joint involvement in the fever group. Therefore, arthritis affecting only one knee and polyarticular arthritis were identified as risk factors for AGA–fever. The inflammatory response is stronger in the knee joint than in other joints, which may be attributed to MSU stimulation of knee synovial cells during an acute episode of knee gout [15], releasing various cytokines that promote an acute systemic inflammatory response [16]. The knee joint, one of the large joints in the body, can release more interleukin (IL)-1, IL-6, and tumour necrosis factor-alpha (TNF-*α*) than smaller joints such as the finger joint, leading to a strong inflammatory response and, consequently, fever [17]. Deposition of urates in the knee cavity causes damage to structures within the joint cavity; stimulates synovial congestion and hyperplasia, leading to activation of inflammatory vesicles; and triggers aseptic inflammation of the synovial membrane within the knee cavity. Some patients with concomitant gouty arthritis of the knee and fever have significantly elevated blood and inflammatory parameters, and synovial fluid examination shows a significant increase in the number of white blood cells, which can easily be misdiagnosed as septic arthritis and treated with antibiotics. In this study, there is a very severe inflammatory reaction during the acute onset of gouty arthritis of the knee joint.

As gout progresses, the number of affected joints increases [8], and some patients may develop a fever ^[18]^. In this study, 11.9% (20/167) of patients had multiple-joint involvement. The involvement of multiple joints usually leads to a stronger inflammatory response, resulting in fever ^[13, 19]^. An acute attack of chronic gout with fever may manifest as noninfectious systemic inflammatory response syndrome, with no evidence of an associated infection ^[19]^. Gout is a multifactorial autoinflammatory disease [12], whereas fever is a prominent feature of many autoinflammatory diseases [16]. This study indicates that patients with multiple-joint involvement are predisposed to fever, which is consistent with the findings of previous studies^[19]^.

In this study, the proportion of elderly patients (age, ≥65 years) was higher in the fever group than in the non-fever group. Older patients with gout are more likely to develop a fever than young and middle-aged patients [13]. Fever in older patients with gout may often be caused by gout-related symptoms [12, 13]. In a study, monocytes from stable patients with gout were stimulated with MSU, and IL-1*β* production in these monocytes was found to increase with the age of patients, suggesting an increased innate immune response to MSU and enhanced formation of “reactive“ MSU (or both) during acute gout attacks in elderly patients, which eventually induces fever. Gout attacks are associated with fever in up to 50% of elderly patients [13]. Gout often occurs in the knee joint in elderly patients ^[20]^. On the one hand, most elderly patients have hyperosteogeny, cartilage strain, and a higher predisposition to urate accumulation in the joints. The deposited urate can accelerate the onset and progression of osteoarthritis and lead to destruction and deformity of bones and joints. When elderly patients with gout present with single knee pain accompanied by fever, the possibility of gouty arthritis of the knee should be considered. If there are no significant risk factors for septic arthritis (i.e. no history of trauma or other infections) in elderly patients with single knee pain, NSAIDs or hormones can be used, and indicators such as white blood cell counts and CRP levels should be closely monitored. A significant decrease in these indicators can confirm the presence of acute gout-induced fever, which reduces the use of unnecessary antibiotics. Because elderly patients have more comorbidities and use a wide variety of medications, prompt identification of the cause of fever and targeted treatment can reduce their medication burden. In patients with chronic gout, recurrent joint attacks may induce systemic inflammatory response syndrome, such as fever ^[19]^. In this study, multivariate logistic regression analysis revealed that elevated CRP levels and VAS scores were independent risk factors for AGA–fever.

This study has several limitations. This study was retrospective and had limited sample size and a single-centre design. The unavailability of the clinical data of some patients might have led to unexpected biases. Moreover, we did not consider the duration of AGA–fever and time of occurrence and duration of the acute phase of gout. Therefore, further prospective studies with larger sample size are warranted to confirm the findings of this study and assess the prognostic and treatment implications of fever in patients with AGA.

## 5. Conclusion

Patients with AGA–fever have more severe pain and more intense inflammatory responses and hence require stronger anti-inflammatory and analgesic drug therapy. In particular, elderly patients with gout and those with arthritis of the single knee or polyarthritis are more likely to develop a fever. Elevated CRP levels and VAS scores are independent risk factors for AGA–fever. Gouty arthritis should be considered if patients with hyperuricemia present with fever and pain in multiple joints or acute pain in the knee. If systemic anti-infective therapy is ineffective in patients with unexplained fever or arthralgia without evidence of infection, they should be carefully queried regarding their past medical history, a detailed physical examination and with dual-energy CT should be performed to determine the presence of gout. In addition, careful identification and management of AGA-caused fever and reduction in antibiotic abuse may help to improve therapeutic efficacy.

## Figures and Tables

**Figure 1:** Multivariate logistic regression analysis. ^∗^*P* < 0.05, ^∗∗^*P* < 0.01.

**Figure 2:** Multivariate logistic regression analysis. ^∗^*P* < 0.05, ^∗∗^*P* < 0.01.

**Table 1:** Degree of fever in 52 patients with AGA.

Factor	Data	Number of cases	Proportion of cases (%)
Low-grade fever	37.3–38°C	27	51.9
Moderate-grade fever	38.1–39°C	23	44.2
High-grade fever	>39.1°C	2	3.9
PCT levels	<0.5*u*g/L	52	100

**Table 2:** Comparison of the clinical characteristics of patients in the fever and non-fever groups.

Indicators	Fever group (*n* = 52; M [Q1, Q3])	Non-fever group (*n* = 115; M [Q1, Q3])	OR	95% CI	*P* value
Sex (men/women)	47/5	107/8	0.70	0.21–2.26	0.553
Age in (years)	63 (40, 73)	57 (38, 67)	—	—	0.148
Disease course (year)	5 (2, 10)	6 (3, 10)	—	—	0.830
White blood cell count (10 ^ 10^9^/L)	8.9 (6.8, 10.4)	7.1(5.8, 9.0)	—	—	0.005
Neutrophil proportion (%)	78.9 (68.1, 84.9)	67.6 (61.0, 75.2)	—	—	0.001
VAS scores	3 (3, 3.5)	2 (2, 3)	—	—	0.001
CRP levels (mg/L)	77 (34, 111)	12 (6, 44)	—	—	0.001
ESR (mm/h)	43 (27, 57)	26 (14, 41)	—	—	0.001
UA levels (*μ*mol/L)	542 (354, 605)	490 (374, 582)	—	—	0.541
Body mass index (kg/m^2^)	25 (24, 27)	26 (24, 29)	—	—	0.041
Age ≥65 years (*n* [%])	25 (48.1)	33 (28.7)	0.44	0.22–0.85	0.016
Renal insufficiency (*n* [%])	18 (34.6)	34 (29.6)	0.79	0.40–1.59	0.514
Hypertension (*n* [%])	29 (55.8)	56 (48.7)	0.75	0.39–1.45	0.397
Type 2 diabetes mellitus (*n* [%])	11 (21.2)	17 (14.8)	0.65	0.28–1.50	0.310
Cardiovascular diseases (*n* [%])	9 (17.3)	14 (12.2)	0.66	0.27–1.65	0.373
NSAID (*n* [%])	37 (71.2)	83 (72.2)	1.05	0.51–2.17	0.892
Oral hormone therapy (*n* [%])	10 (19.2)	13 (11.3)	0.53	0.22–1.32	0.169
Oral colchicine therapy (*n* [%])	18 (34.6)	48 (41.7)	1.35	0.68–2.67	0.383
Betamethasone injection (*n* [%])	38 (73.1)	54 (47.0)	0.32	0.16–0.67	0.002
NSAIDs combined with betamethasone (*n* [%])	25 (48.1)	35 (30.4)	0.47	0.24–0.92	0.028

**Table 3:** Comparison of the involved joints between the fever and non-fever groups.

Involvement pain sites	Fever group (*n* = 52)	Non-fever group (*n* = 115)	OR	95% CI	*P* value
Single knee joint (*n* [%])	20 (38.5)	26 (22.6)	2.14	1.05–4.35	0.034
Ankle joint (*n* [%])	7 (13.5)	26 (22.6)	0.53	0.22–1.32	0.169
First toe joint (*n* [%])	3 (5.8)	29 (25.2)	0.18	0.53–0.63	0.003
Back of the foot (*n* [%])	4 (7.7)	10 (8.7)	0.87	0.26–2.93	0.828
Finger joint (*n* [%])	1 (1.9)	5 (4.3)	0.43	0.05–3.79	0.436
Wrist joint (*n* [%])	3 (5.8)	5 (4.3)	1.35	0.31–5.86	0.690
Shoulder joint (*n* [%])	1 (1.9)	3 (2.6)	0.73	0.07–7.20	0.788
Elbow joint (*n* [%])	1 (1.9)	2 (1.7)	1.11	0.10-12.5	0.934
Multiple joints (*n* [%])	11 (21.2)	9 (7.8)	3.16	1.22–8.16	0.014

**Table 4:** Multivariate logistic regression analysis.

Indicators	*β*-Value	Standard deviation	Wald value	*P* value	OR	95% CI
CRP levels	0.014	0.005	7.707	0.005	1.014	1.004–1.025
ESR	0.008	0.011	0.455	0.500	1.008	0.986–1.030
VAS scores	0.523	0.211	6.139	0.013	1.686	1.115–2.549
White blood cell counts	0.046	0.079	0.336	0.562	1.047	0.897–1.222
Neutrophil proportion	0.017	0.020	0.732	0.392	1.017	0.978–1.059
UA levels	0.002	0.002	1.664	0.197	1.002	0.999–1.005
Age of ≥65 years	-0.566	0.442	1.643	0.200	0.568	0.239–1.350
Single knee joint	0.120	0.501	0.058	0.810	1.128	0.422–3.012
Multiple joints	-0.407	0.620	0.432	0.511	0.666	0.198–2.241
First toe joint	0.801	0.732	1.197	0.274	2.228	0.530-9.361

## Data Availability

The research data used to support the findings of this study are available from the corresponding author upon request.

## Additional Points

*Key Summary Points.* (1) Patients with fever symptoms of acute gout are mainly low-grade fever. (2) Acute knee gout and polyarticular gout were more likely to have fever. (3) Patients with acute gout with fever symptoms, stronger anti-inflammatory and analgesic drugs should be recommended. (3) Elevated CRP levels and VAS scores are independent risk factors for acute gouty arthritis with fever.
